# Feature Fusion-Based Improved Capsule Network for sEMG Signal Recognition

**DOI:** 10.1155/2022/7603319

**Published:** 2022-01-21

**Authors:** Wanliang Wang, Wenbo You, Zheng Wang, Yanwei Zhao, Sheng Wei

**Affiliations:** ^1^College of Computer Science and Technology, Zhejiang University of Technology, Hangzhou 310023, Zhejiang, China; ^2^College of Modern Information Technology, Zhejiang Institute of Mechanical Electrical Engineering, Hangzhou 310053, Zhejiang, China

## Abstract

This paper proposes a feature fusion-based improved capsule network (FFiCAPS) to improve the performance of surface electromyogram (sEMG) signal recognition with the purpose of distinguishing hand gestures. Current deep learning models, especially convolution neural networks (CNNs), only take into account the existence of certain features and ignore the correlation among features. To overcome this problem, FFiCAPS adopts the capsule network with a feature fusion method. In order to provide rich information, sEMG signal information and feature data are incorporated together to form new features as input. Improvements made on capsule network are multilayer convolution layer and e-Squash function. The former aggregates feature maps learned by different layers and kernel sizes to extract information in a multiscale and multiangle manner, while the latter grows faster at later stages to strengthen the sensitivity of this model to capsule length changes. Finally, simulation experiments show that the proposed method exceeds other eight methods in overall accuracy under the condition of electrode displacement (86.58%) and among subjects (82.12%), with a notable improvement in recognizing hand open and radial flexion, respectively.

## 1. Introduction

Surface electromyogram (sEMG), an electrical signal generated on skin surface during muscle contraction, contains rich information about muscle activity and can be used to identify the subject's action intention [1]. Thus, it is commonly used in rehabilitation, intelligent bionics, and human–computer interaction [2]. In practical applications, accurate and fast classification of signals is the basic prerequisite. Since sEMG signal is susceptible to factors such as physiological state of the subject or physical characteristics of the device, accuracy of classification algorithms will vary from person to person or time to time. As a consequence, algorithms with higher accuracy under different conditions are in urgent need.

In early stages of sEMG recognition, feature extraction is often applied to time windows, and feature data is sent to machine learning models, such as support vector machine (SVM), random forest (RF), and linear discriminant analysis (LDA) [3–5]. However, methods as mentioned are already clearly defined, which means there are only limited ways to improve classification performance. That is, adjust hyperparameters or change the combination or order of features. And the effects of those methods are not that satisfying.

With the development of deep learning, more problems in fields like image processing or speech recognition are solved in a better way. Recently, deep learning methods are adopted in sEMG recognition, as deep learning models have strong abilities of feature extraction and model fitting [6]. Geng et al. [7] put forward the concept of sEMG image, which means the conversion from multichannel signal into images and completed the gesture recognition experiments based on convolution neural network (CNN), achieving the accuracy of 65.1% of NinaPro DB1 dataset. Chen et al. [8] designed a deep CNN model and tested it on NinaPro DB5 dataset, where the signal was processed with continuous wavelet transform, thus reducing the number of parameters and achieving the accuracy of 69.62%, 67.42, and 61.63% for three subsets. Barron et al. [9] proposed to classify sEMG signals of different subjects by using recurrent neural network (RNN), which is higher in classification accuracy of 79.7% in their own dataset.

Although the recognition performance is gradually improving with the help of deep learning, classification of sEMG signal still faces challenges [10]. On the one hand, deep learning methods are usually applied to images and their appliance in one-dimensional signal is limited. To adapt to various models, sEMG signal is often transformed into two-dimensional data, like sEMG images [7]. For sEMG images that vary linearly from sEMG signal or sequences cut from sEMG signal [11], they contain a lot of redundant information and cannot reflect the characteristics in frequency domain or time-frequency domain well. On the other hand, pooling operation, which is commonly applied to downsample features and decrease parameters, suffers from information loss. Meanwhile, it is impossible to discover the potential links between features using convolution only, the most commonly used method to extract features from input. Such lost information and undiscovered correlation among features may contain key information for certain gestures and help to solve the problem where current algorithms fail to achieve satisfying results. Those problems may occur when there are small differences in the muscles contracted for some gestures or too many gestures to be recognized.

To address the previously mentioned challenges, this paper proposes an improved capsule network (CapsNet) method based on feature fusion. Using fused features instead of sEMG images or sequences, the complexity of the model is reduced. Moreover, the structure of capsule network is improved to make the network more suitable for the characteristics of sEMG signals. The proposed method has achieved good results on the experiments of electrode displacement and different subjects respectively. The main contributions of this paper are summarized as follows.

First, this research proposes a new method to generate features by feature fusion. Fused features not only make up for information loss during feature extraction but also enable the model to explore the potential links between features.

Second, the original convolution layer is replaced with multilevel convolution layer, so that features of different layers and angles are concatenated to enrich the information for subsequent layers, and thus, the model is deepened the broadened.

Third, FFiCAPS modifies the squash function to suit the recognition of sEMG signal by adopting e-Squash. The effects of squash function will vary with datasets. The e-Squash enables higher growing rate as the capsule length grows to a certain extent to strengthen the model's sensitivity.

The structure of this paper is as follows. The second section introduces the improved capsule network framework based on feature fusion, the third section carries out relevant experiments and verification on the proposed method, and the fourth section summarizes the full text.

## 2. The Proposed Method

In this section, we first introduce the method to combine sEMG signal and feature data. Then, we introduced the structure of CapsNet and proposed improvements are explained in detail.

### 2.1. Feature Fusion Method

This method mainly consists of two stages. The first one is dealing with feature data and sEMG signal information, while the other one is stacking them together to form new abstract feature maps. The detailed process is shown in Figure 1.

Suppose *m* features are extracted from one channel of sEMG window of length *w*, and the feature vector *f* can be expressed as

(1) $$\begin{array}{c} f=\left[1,x_{1},x_{2},\ldots ,x_{i},\ldots ,x_{m}\right], \end{array}$$

where *x*_*i*_ denotes a single feature and 1 is added to maintain original features. Here, *m* equals 14 and *w* equals 300. The detailed description of features is shown in Table 1 in Section 3.2.

Feature vectors are combined according to the rules of matrix multiplication and transformed into feature maps. The calculation process is shown as follows:

(2) $$\begin{array}{c} F=G\left(\mathrm{\alpha *}{\left(f^{T}\times f\right)}^{\beta }\right), \end{array}$$

where × denotes matrix multiplication, *α* and *β* are conversion parameters, both equal to 0.5, G is the sigmoid function shown in (3), and *F* represents the feature map that contains fused abstract features.

(3) $$\begin{array}{c} G\left(\theta \right)=\text{sigmoid}\left(\theta \right)=\frac{1}{1+e^{-\theta }}, \end{array}$$

where *θ* is the only input of the sigmoid function G that is applied to restrict the output to range (0, 1).

As sEMG signal contains rich information, it is considered to be fused into feature maps to make up for information loss. Each sEMG window of length *w* is cut into *n* segments according to the length *l*. The parameters *n* and *l* meet the demand of

(4) $$\begin{array}{c} \text{dif}=\min\left(\left|n-l\right|\right)\\ s.t\;n*l=w, \end{array}$$

where *dif* means the minimum absolute value of difference between *n* and *l*. Therefore, *n* and *l* are equal to 15 and 20, respectively. These segments were stacked to form a sEMG matrix of dimension *n* × *l*.

Convolutions with different kernel sizes are applied to fuse the processed sEMG signal and feature matrix as their shapes are different. In this paper, 256 convolutions of kernel size 3 × 8 and of 3 × 3 are used to deal with sEMG matrix and feature matrix, respectively, using for both a stride equal to 2. Following the previously mentioned operations, feature maps generated from feature data and sEMG signal are concatenated on the channel, which is often the method to fuse feature maps. Moreover, 1 × 1 convolution with 256 channels is introduced to strengthen the expressiveness of network. Finally, as features of different sources vary from amplitudes, Min-Max normalization has to be done before training, as it is shown in the following equation:

(5) $$\begin{array}{c} X_{\text{norm}}=\frac{X_{i}-X_{\min}}{X_{\max}-X_{\min}}, \end{array}$$

where *X*_*i*_ is a single data in a feature map, *X*_min_ means the minimum value in the feature map, *X*_max_ means the maximum value in the feature map, and *X*_norm_ means the normalized output. The normalization operation accelerates the process of gradient descent and enables features originated from sEMG signal and feature data to make the same contribution to results.

### 2.2. Improved CapsNet

Capsule network is a model with vectors as basic blocks [11], which not only reflects whether a certain feature is present or not but also has the ability to uncover the potential connections between features. The improved capsule network replaces the traditional single convolutional layer with a multilevel convolutional layer and squash function with an e-Squash function on original capsule network. The specific structure is shown in Figure 2.

#### 2.2.1. CapsNet

Capsule network is a deep learning model based on capsules. A capsule consists of multiple neurons, and each neuron represents a certain attribute of a specific entity in the input. The vector length of capsule ranges from [0, 1), with larger lengths representing higher possibility of a certain entity to exist. And the vector direction suggests the instantiated parameter. Different from CNN, capsule network abandons pooling layer and adopts dynamic routing mechanism instead to connect capsules at different levels, thus achieving robust and reliable results [14]. The process of dynamic routing can not only obtain the spatial relationship between the whole and parts but also route the information between capsules by strengthening the connection between capsules, so that capsules at different levels can achieve high consistency [15]. The specific process is shown in Figure 3.

As shown in Figure 3, *u*_*i*_ is the output of primary capsule *i*, and it is multiplied by transformation matrix *W*_*ij*_ to obtain prediction vector *û*_*j|i*_. All prediction vectors *û*_*j|i*_ are multiplied and accumulated by their coupling coefficients *c*_*ij*_, and then, the output is mapped to a restricted range by squash function to obtain the output *v*_*j*_ of action capsule *j*. The formula of calculation process is as follows:

(6) $$\begin{array}{c} {\text{û}}_{j|i}=W_{ij}u_{i}, \end{array}$$

where *W*_*ij*_ is the transformation matrix that connects primary capsule *i* and action capsule *j*, and *û*_*j|I*_ is the prediction vector of the *i*-th primary capsule for the *j*-th action capsule. The coupling coefficients *c*_*ij*_ is calculated as

(7) $$\begin{array}{c} c_{ij}=\frac{\exp\left(b_{ij}\right)}{\sum_{k}\exp\left(b_{ik}\right)}, \end{array}$$

where *c*_*ij*_ is the coupling coefficient between primary capsule *i* and action capsule *j*. The sum of all coupling coefficients between primary capsule *i* and all action capsules is 1. For the value of the coupling coefficient *c*_*ij*_, it is determined by the prior probability *b*_*ij*_ that the primary capsule *i* is coupled to action capsule *j* and the initial value of *b*_*ij*_ is set to 0. Prior probability *b*_*ij*_ will be updated in the subsequent iterations to update the coupling coefficient *c*_*ij*_.

(8) $$\begin{array}{c} s_{j}=\sum_{i}c_{ij}{\text{û}}_{j|i}, \end{array}$$

where *s*_*j*_ is the weighted sum of all prediction vectors *û*_*j|I*_ and is fed into the squash function.

(9) $$\begin{array}{c} v_{j}=\frac{{\left\|s_{j}\right\|}^{2}}{1+{\left\|s_{j}\right\|}^{2}}\frac{s_{j}}{\left\|s_{j}\right\|}, \end{array}$$

where *v*_*j*_ is the output of action capsule *j*. In order to restrict the length of the vector to [0,1) to represent the probability of entity existence, a nonlinear squash function is used to reduce the vector size to 0 for shorter vector lengths and to slightly less than 1 for longer vector lengths.

(10) $$\begin{array}{c} b_{ij}=b_{ij}+{\text{û}}_{j|i}•v_{j}. \end{array}$$

Before calculating new coupling coefficient *c*_*ij*_, value of the prior probability *b*_*ij*_ is updated and the product of predicted vector *û*_*j|i*_ and output vector *v*_*j*_ is added to the original base. A larger value of the product represents a closer orientation of a lower level capsule to a higher level capsule and a larger coupling coefficient between the capsules. In this way, the coupling between two similar capsules will be tighter during iterations.

For each action capsule, a separate margin loss function is used to calculate the loss. The total loss of the network is equal to the sum of the losses of all action capsules.

(11) $$\begin{array}{c} L_{k}=\sum_{k=1}^{N}\left(T_{k}\max{\left(0,m^{+}-\left\|v_{k}\right\|\right)}^{2}+\lambda \left(1-T_{k}\right)\max{\left(0,\left\|v_{k}\right\|-m^{-}\right)}^{2}\right), \end{array}$$

where value of *T*_*k*_ is either 0 or 1. The value of 1 for *T*_*k*_ means that the entity represented by this action capsule exists and vice versa. For hyperparameters m^+^ and m^−^, they are set to 0.9 and 0.1, which mean loss is 1 if the possibility is less than 0.1 and 0 if the possibility is greater than 0.9, respectively. Weight parameter *λ* serves to determine the influence of predicting an incorrect label and it is set to be 0.5. The number of iterations for dynamic routing is 3.

#### 2.2.2. Multilevel Convolution

Original capsule network extracts features by using a convolution layer and then feeds the output to subsequent layers.

Instead of a single convolution layer, a multilevel convolutional layer is proposed, where convolutional kernels of different scales are adopted to extract information in a multiscale and multiangle manner. To be specific, we adopt 256 convolutions of kernel size 3 × 3 and 256 convolutions of kernel size 5 × 5 and stack the feature maps gained by these operations on the channel. So as not to miss the information of the previous layer, the output of previous layer is stacked directly with obtained feature maps.

As stacking on the channels brings an increase in the number of channels and parameters, a bottleneck layer, 256 convolutions with a kernel size of 1 × 1, is introduced to reduce the number of channels and parameters and shorten the calculation time.

#### 2.2.3. e-Squash

The squash function of capsule network can be divided into two parts according to their functions: one is to find the unit vector of the input vector, and the other is to compress the length of this unit vector to [0, 1) by a nonlinear function, thus realizing the activation function of the capsule. Improvements are made for the latter part.

The original squash function grows rapidly at the starting stage, and even if the length of a particular capsule is small, it is still able to obtain a relatively large activation value. As the length of the capsule grows, the function value slowly approaches to 1. In order to suit the characteristics of sEMG signal, the growth rate of the function needs to be appropriately changed. However, too large growth rate in the initial stage is likely to lead to too large activation values. The probability of the existence of the entity represented by the capsule will be amplified due to the sensitivity of dynamic routing, leading to a decrease in classification accuracy. Therefore, the squash function needs to be improved to maintain its growth rate at the initial stage and to enhance the function growth rate in the subsequent stages to find out valid information.

Based on the previously mentioned discussion, an improvement for the nonlinear function part of the Squash function was proposed in this paper and the new function is called e-Squash as follows:

(12) $$\begin{array}{c} v_{j}=\left(1-e^{-{\left\|s_{j}\right\|}^{{}^{2}}}\right)\frac{s_{j}}{\left\|s_{j}\right\|}. \end{array}$$

The function curve is almost identical to that of the original Squash function when the vector length is small and rises faster than the original Squash function after the vector length reaches a certain value, which improves the sensitivity of the response and is eventually stable.

## 3. Experiments and Analysis

### 3.1. The sEMG Dataset

The sEMG dataset was acquired using ELONXI device developed by the team at University of Portsmouth, UK [16]. This device supports a maximum of 16 channels with a sampling resolution of 24 bits and a sampling frequency between 1000 Hz and 2000 Hz. In this dataset, 16 channels with a sampling frequency of 1000 Hz mode were selected, and the filtered signal was obtained using the filter that was built within this system. In specific, the signal passed through a band-pass filter (20–500 Hz), and then, a band-stop filter at 50 Hz is used to remove the power line interference.

Eight subjects' sEMG signals were collected for six different time periods, and the same five gestures were collected for each time period. The movements are hand closed (HC), hand open (HO), radial flexion (RF), wrist flexion (WF), and wrist extension (WE). To simulate different situations, three time periods are executed in the morning and the rest three time periods are in the afternoon, with the equipment worn once in the morning and once in the afternoon, respectively. In order to reduce the influence of muscle fatigue, all subjects rested for 10 seconds between every two movements and 30 minutes between every two time periods.

### 3.2. Preprocessing and Feature Extraction

Considering that sEMG is a period of time series, window analysis is applied to preprocess the signal. This method mainly involves two parameters, namely, the length of the window and the increment interval. The length of window represents the unit length of signal processing, which directly affects the recognition accuracy. The incremental interval *τ* affects response time of the system, which is a key factor for the application of sEMG signals. The window cutting method is shown in Figure 4, where *w* is the window length and *τ* is the increment interval. Here, *w* equals 300 and *τ* equals 50.

As the purpose of this paper is to explore a new method for sEMG recognition instead of feature selection, feature selection is not discussed in detail, and 14 commonly used features are selected, provided by time domain and frequency domain.

In Table 1, *S*_*i*_ represents the signal of a window. *S*_*f*_ represents the spectrum obtained by Fast Fourier transform of the window, and P(*S*_*f*_) represents the power spectrum intensity obtained by calculating the square of the norm of spectrum *S*_*f*_. The features used in the experiment are shown in Table 1.

### 3.3. Recognizing sEMG Signal under Different Conditions

In current applications of sEMG signal, there are two main difficulties getting in the way. First, there are differences in the position of the sEMG acquisition device each time it is worn, resulting in different positions of the electrodes corresponding to the muscles. Besides, it is also common for sEMG acquisition device to shift the position due to external forces or other factors in actual use. Second, sEMG signals have large differences in values between different people, so it is necessary to dig deeply into the universal features of sEMG signals. To address the previously mentioned issues, two experiments are designed in this paper to test the performance of the proposed method in case of electrode displacement and different people.

The experimental environment is Windows 10, CPU i7-9750H, GPU 1660Ti, and tensor flow. Structural parameters of network are shown in Table 2.

#### 3.3.1. Recognizing sEMG under Electrode Displacement

The specific situation of electrode displacement is as follows: sEMG from one subject was repeatedly collected three times in the morning as the training set, and the data collected in the afternoon was used as the testing set. Each subject wore the device once in the morning and once in the afternoon, thus simulating the case of electrode displacement. The experiment was set with a batch-size of 32, and Adam algorithm was used to optimize the loss. Different methods are tested to see whether the proposed method works or not. The results are displayed in Table 3.

FE means feature extraction, and FF means feature fusion. Bolded fonts stand for best performance in each column.

For traditional machine learning methods SVM and RF, which used extracted features as the input, they have excellent results in distinguishing certain actions, reaching 100% accuracy in action WE and WF, but fail to reach high accuracy in action HO and HC. Thus, the overall performance is not that satisfying. It shows traditional machine learning methods have some defects to some extent.

CNN is a commonly used model for deep learning. In this experiment, sEMG signal, extracted features, and fused features are used as inputs for comparison.

Using sEMG signal as input of CNN, the accuracy is the lowest among all three inputs because sEMG signal contains a lot of redundant information and can hardly reflect the features of other domains. In particular, the accuracy of action HO and RF are less than 15%. The accuracy of CNN with features as input can hardly recognize action HO, indicating that it is difficult to obtain the information characterizing action HO. It is worth noting that overall accuracy of using the fused features is the highest among three inputs, and it performs relatively better on action HO than discrete features or original signal, though it is still at a low level, indicating that this feature fusion method can characterize some of the properties of action HO. For DNN which uses extracted features as input, it has a low overall accuracy due to poor performance on action HO.

TDACAPS, CAPS, and FFiCAPS are models based on capsule networks. The difference is that TDACAPS adds attention mechanism to capsule network, and FFiCAPS makes improvements to the structure of capsule network. Besides, TDACAPS takes extracted features as input, while CAPS and FFiCAPS takes fused features as input. FFiCAPS improves the convolution layer and squash function of the capsule network compared with CAPS, thus making the capsule network more suitable for the recognition of sEMG signals. The overall accuracy of FFiCAPS is higher than that of CAPS and TDACAPS and is the highest among all methods. More importantly, FFiCAPS achieves the best accuracy of 80.61% for action HO, which indicates that the proposed method can indeed mine the information characterizing action HO.

It is worth noting that no method has accuracy higher than 85% for HO. Some gestures trigger similar changes in sEMG signal to others and are therefore difficult to classify accurately. This may account for poor classification performance for HO. Comparing three types of inputs, sEMG signal, extracted features, and fused features, the experimental results illustrate the validity of proposed feature fusion method. Meanwhile, it can also be concluded that improvements on CapsNet are suitable for sEMG signal recognition, considering FFiCAPS achieves the highest accuracy of 80.61%.

In addition, the accuracy and loss performance of each method is compared in this section.  Figure 6(a) shows the curve of testing accuracy of each method, and Figure 6(b) shows the loss curve of each method. From Figure 6(b), it can be seen that the loss of each method decreases and tends to be smooth with the increase of iterations. And the test accuracy in Figure 6(a) increases gradually with the increase of iterations. Compared with CNN and DNN, the accuracy of methods based on capsule network lags behind at first, but it gets higher after a certain number of iterations. Among TDACAPS, CAPS + FF, and FFiCAPS, FFiCAPS reaches the highest accuracy in the end.

#### 3.3.2. Recognizing sEMG from Different People

To recognize sEMG signals from different people, it is required that the classifier should be able to mine general features from sEMG and find out the link between these features and gestures from subjects. The experiment was set with a batch size of 16, and Adam algorithm was used to optimize the loss. Different methods are tested to see whether the proposed method works. The results are displayed in Table 4.

It is demonstrated that traditional machine learning methods perform well in this experiment with overall accuracy higher than 70%. RF even achieves the highest accuracy in distinguishing action WE, though its accuracy for action WF is relatively low. As for SVM, it performs well in action WF but does not get high accuracy in action HO. Therefore, the machine learning approach has some advantages when it comes to robustness of the algorithm or mining general characteristics of sEMG signal. However, the recognition accuracy still needs to be improved, which does not reach 80%.

The accuracy of CNN with sEMG signal as input for different subjects is only 69.27%, the lowest of all methods, while the accuracy with extracted features or fused features as input is above 75%. Moreover, the accuracy of the fused features is 0.27% higher than that of extracted features, which illustrates the effectiveness of the feature fusion method proposed in this paper. Although the overall improvement seems small, it does help to discover the valid information for action WF compared with CNN with extracted features. It can be seen that CNN with sEMG signal as input reaches the highest accuracy in recognizing action WF and CNN with extracted features only get 19.91%. For CNN with fused features as input, it is 33.66% higher than that of CNN with extracted features as input, which proves that the proposed method enriches the input information. DNN achieves the best accuracy on action HC and WE but does not perform well on action HO and RF, resulting in its total accuracy lower than 80%.

The accuracy of capsule networks was generally higher than that of CNNs, indicating that capsule networks can reduce the loss of information and facilitate the mining of general features of sEMG signal. Among the three methods based on capsule network, TDACAPS achieves the highest accuracy on action HO. FFiCAPS achieves the highest overall accuracy, which is 6.2% higher than CAPS and a bit higher than TDACAPS. Moreover, the performance of FFiCAPS is the best on gesture HC, RF, WE, and WF among three methods based on capsule network, and it reaches the top accuracy on gesture RF among all methods.

Besides, the performance of all methods in accuracy and loss is compared in this section. In Figure 7(a), it can be seen that accuracy of all methods gradually increases in spite of some ups and downs. Compared with CNN and DNN, methods based on capsule network are left behind when iteration is less than 10 but catch up with other methods later. As for loss in Figure 7(b), all methods decrease gradually, and there is no obvious lag in methods based on capsule network.

#### 3.3.3. Testing for Different Squash Functions

Squash function is a crucial component of capsule network. So as to test e-Squash, various squash functions are compared in this section. The squash function equations and curves are shown in Table 5 and Figure 8, respectively. The effectiveness of the proposed e-Squash function is verified by experiments and the results are shown in Table 6.

In the case of electrode displacement, all methods using e-Squash obtain a higher accuracy than those using the original Squash function. As for FFiCAPS, four different squash functions show an improvement in overall accuracy compared with the original Squash function. e-Squash proposed in this paper shows the largest improvement of 4.84% followed by strict-Squash, indicating that e-Squash function is beneficial for improving accuracy.

In the case of different subjects, CAPS with e-Squash reaches a higher accuracy, while TDACAPS does not fit well with e-Squash and perform worse than original model. Perhaps, the combination of spatial attention and e-Squash fails to focus on valid information of abstract features and tend to cause overfitting. For FFiCAPS, the differences in overall accuracy are not significant. HSquash is slightly better than the original Squash function. Squash-4 and strict-Squash perform worse than the original Squash function. And e-Squash has the best result, with a 4.05% improvement compared with the original Squash.

#### 3.3.4. Computational Resources Consumed

In this section, training time and recognition time for all methods under the case of electrode displacement and different subjects are compared in Table 7.

In terms of computing resources, SVM and RF only consume little time to train and recognize. For models based on CNN or DNN, their consumption of time is more than machine learning methods, but their accuracy is higher than that of SVM and RF. The models that have the largest time consumption are models based on capsule network, as they do not apply pooling operations and dynamic routing requires a large number of training parameters. But they make improvement on overall performance and the recognition time is still acceptable, which meets the requirement for time delay.

## 4. Conclusions

In this paper, we propose a framework named FFiCAPS, which consists of a new method of generating fused features and capsule network with modifications. Our method is able to capture the correlation among extracted features and decrease the information loss.

The effectiveness of the proposed method is verified by two experiments that are under the case of electrode displacement and under different subjects. In electrode displacement, the accuracy for hand open is particularly poor. Among all competing methods, our method had the highest accuracy of 80.61% for hand open, which is much higher than that of models based on convolution neural network. Besides, FFiCAPS also achieved the best overall accuracy in electrode displacement, which illustrates the effectiveness of proposed method. When it comes to different subjects, the proposed method achieved the highest accuracy, though overall improvement compared with the second best accuracy is small. However, it is true that our method achieved the highest accuracy on four gestures out of five among three models based on capsule network and performed the best on radial flexion. This proves that in robustness our method also has some advantages.

The method proposed in this paper can meet the realistic requirements of both time delay and accuracy, but it still needs to be improved in terms of computational efficiency. Dynamic routing consumes a large amount of computational resources, so the next goal is to optimize the dynamic routing mechanism, improve the computational efficiency, and further enhance the performance of gesture recognition.

## Figures and Tables

**Figure 1:** The feature fusion method. The sEMG signal is cut and stacked, and feature data is transformed into two-dimensional feature map. They are concatenated after convolution operations.

**Figure 2:** The structure of proposed FFiCAPS framework. The input is the feature map mentioned in Section 2.1. The main improvement in FFiCAPS is multilevel convolution layer and e-Squash function.

**Figure 3:** Dynamic routing mechanism. Capsules at different levels are connected through this mechanism.

**Figure 4:** Window analysis method. sEMG signal is cut into time windows of the same length (w) with the same time interval *τ*.

**Figure 5:** The process of feature fusion method. Detailed parameters and operations are shown.

**Figure 6:** The testing accuracy and loss of different methods under electrode displacement. (a) The accuracy. (b) The loss.

**Figure 7:** The testing accuracy and loss of different methods under different people. (a) The accuracy. (b) The loss.

**Figure 8:** The squash function curves of five different squash functions.

**Table 1:** Features selected in the experiment.

Feature	Name	Description	Equation
*x*_1_	RMS [12]	Relates to amplitude changes	$\sqrt{1/w*\sum_{i=1}^{w}S_{i}^{2}}$
*x*_2_	MAV [12]	Reflection on muscle contraction levels	1/*w∗*∑_*i*=1_^*w*^|*S*_*i*_|
*x*_3_	WL [12]	Accumulated wavelength	∑_*i*=1_^*w*−1^|*S*_*i*+1_ − *S*_*i*_|
*x*_4_	ZC [12]	Times that sEMG signal crosses zero in amplitude	∑_*i*=1_^*w*−1^[sgn(*S*_*i*_•*S*_*i*+1_)∩|*S*_*i*_ − *S*_*i*+1_|≥ε]
*x*_5_	DASDV [12]	The standard deviation value of wavelength	$\sqrt{1/\left(w-1\right)*\sum_{i=1}^{w-1}{\left(S_{i+1}-S_{i}\right)}^{2}}$
*x*_6_	LOG [12]	Estimation of muscle contraction force	exp(1/*w∗*∑_*i*=1_^*w*^*S*_*i*_)
*x*_7_	SSI [12]	Energy of the signal	∑_*i*=1_^*w*^*S*_*i*_^2^
*x*_8_	TM3 [12]	The third moment of sEMG signal	|1/*w∗*∑_*i*=1_^*w*^*S*_*i*_^3^|
*x*_9_	TM4 [12]	The fourth moment of sEMG signal	|1/*w∗*∑_*i*=1_^*w*^*S*_*i*_^4^|
*x*_10_	TM5 [12]	The fifth moment of sEMG signal	|1/*w∗*∑_*i*=1_^*w*^*S*_*i*_^5^|
*x*_11_	FR [12]	Degree of muscle contraction and relaxation	∫_*LLC*_^*ULC*^*P*(*S*^*f*^)d*S*^*f*^/∫_*LHC*_^*UHC*^*P*(*S*^*f*^)d*S*^*f*^
*x*_12_	IEMG [12]	Estimation of signal power	∑_*i*=1_^*w*^|*S*_*i*_|
*x*_13_	MFMN [13]	Average frequency of sEMG	∫_0_^+*∞*^*S*^*f*^*P*(*S*^*f*^)d*S*^*f*^/∫_0_^+*∞*^*P*(*S*^*f*^)d*S*^*f*^
*x*_14_	MFMD [13]	Median frequency of sEMG	1/2*∗*∫_0_^+*∞*^*P*(*S*^*f*^)d*S*^*f*^

**Table 2:** Structural parameters of improved CapsNet.

Layer	Operation	Kernel/stride	Output/channel	Padding
Input	-	-/-	7 × 7/256	-
ML-Conv	Conv3∗3	3 × 3/1 × 1	7 × 7/256	Y
	Conv5∗5	5 × 5/1 × 1	7 × 7/256	Y
	Concat	-/-	7 × 7/768	-
	Conv1∗1	1 × 1/1 × 1	7 × 7/256	N
PrimaryCaps	Reshape	-/-	7 × 7∗8/32	-
ActionCaps	-	-/-	5/16	-
Class	-	-/-	5/-	-

Besides, detailed process and parameters of feature fusion method are shown in Figure 5.

**Table 3:** Recognition accuracy under electrode displacement.

Method	Gesture recognition accuracy (%)					Overall accuracy (%)
	HC	HO	RF	WE	WF	
SVM + FE [17]	36.41 ± 0.00	3.08 ± 0.00	86.15 ± 0.00	**100** **±** **0.00**	**100** **±** **0.00**	65.13 ± 0.00
RF + FE [18]	65.64 ± 0.00	14.36 ± 0.00	84.10 ± 0.00	**100** **±** **0.00**	**100** **±** **0.00**	78.36 ± 0.00
CNN [19]	**98.72** **±** **1.67**	11.42 ± 8.18	14 ± 9.55	97.79 ± 1.38	90 ± 3.49	63.36 ± 2.31
CNN + FE	81.38 ± 4.24	1.64 ± 1.16	89.64 ± 3.60	99.90 ± 0.31	91.90 ± 0.45	74.03 ± 0.76
CNN + FF	94.56 ± 4.44	35.33 ± 15.32	74.87 ± 10.10	97.85 ± 1.39	85.18 ± 4.42	78.77 ± 1.26
DNN + FE [20]	84.67 ± 3.89	0.50 ± 0.63	92.92 ± 4.15	99.48 ± 0.92	92.31 ± 0.00	75.18 ± 1.25
TDACAPS [21]	97.59 ± 2.62	74.87 ± 15.71	**95.18** **±** **4.42**	98.56 ± 1.82	55.39 ± 16.87	84.77 ± 0.82
CAPS + FF.	98.41 ± 4.27	44.15 ± 9.82	92.51 ± 7.58	99.74 ± 0.77	78.92 ± 6.71	84.04 ± 2.54
∗FFiCAPS	97.74 ± 4.26	**80.61** **±** **8.53**	93.02 ± 5.78	99.74 ± 0.77	55.26 ± 16.92	**86.58** **±** **2.70**

**Table 4:** Recognition accuracy under different people.

Method	Gesture recognition accuracy (%)					Overall accuracy (%)
	HC	HO	RF	WE	WF	
SVM + FE [17]	93.85 ± 0.00	54.19 ± 0.00	50.34 ± 0.00	99.66 ± 0.00	72.74 ± 0.00	74.15 ± 0.00
RF + FE [18]	93.76 ± 0.00	81.45 ± 0.00	53.76 ± 0.00	**100** **±** **0.00**	28.97 ± 0.00	71.59 ± 0.00
CNN [19]	68.42 ± 2.55	50.78 ± 0.56	49.43 ± 1.73	98.85 ± 0.08	**76.82** **±** **1.50**	69.27 ± 0.68
CNN + FE	99.94 ± 0.09	75.38 ± 14.97	80.32 ± 0.81	98.82 ± 1.60	19.91 ± 15.56	75.21 ± 0.44
CNN + FF	88.63 ± 0.17	76.83 ± 3.88	57.05 ± 8.97	99.62 ± 0.77	53.57 ± 17.71	75.48 ± 0.17
DNN + FE [20]	**99.98** **±** **0.05**	75.89 ± 0.68	66.80 ± 0.54	**100** **±** **0.00**	46.79 ± 0.53	78.24 ± 0.15
TDACAPS [21]	98.25 ± 3.89	**84.98** **±** **7.12**	82.48 ± 5.96	98.24 ± 0.62	44.75 ± 5.50	81.90 ± 1.09
CAPS + FF.	98.68 ± 2.29	69.86 ± 4.78	68.94 ± 11.22	99.21 ± 0.78	41.23 ± 4.58	75.92 ± 1.38
*∗*FFiCAPS	98.78 ± 0.56	78.70 ± 5.40	**85.51** **±** **5.78**	99.98 ± 0.05	45.83 ± 3.53	**82.12** **±** **0.90**

FE means feature extraction, and FF means feature fusion. Bolded fonts stand for best performance in each column.

**Table 5:** The equations for different squash functions.

Squash function	Equation
Squash [14]	*v*_*j*_=(‖*s*_*j*_‖^2^/(1+‖*s*_*j*_‖^2^)(*s*_*j*_/‖*s*_*j*_‖))
HSquash [22]	*v*_*j*_=‖*s*_*j*_/4‖^2^/1+‖*s*_*j*_/4‖^2^*s*_*j*_/‖*s*_*j*_‖
Strict-squash [23]	*v*_*j*_=0.69‖*s*_*j*_‖^2^*∗*2^−0.6‖*s*_*j*_‖−1.115^
Squash-4 [24]	*v*_*j*_=‖*s*_*j*_‖^2^/0.5+‖*s*_*j*_‖^2^*s*_*j*_/‖*s*_*j*_‖
e-Squash	*v*_*j*_=(1 − *e*^−‖*s*_*j*_‖^2^^)*s*_*j*_/‖*s*_*j*_‖

**Table 6:** Recognition accuracy of different squash functions.

Methods	Squash function	Under electrode displacement	Under different people
CAPS + FF	Squash [14]	84.04 ± 2.54	75.92 ± 1.38
CAPS + FF	e-Squash	84.68 ± 1.41	76.06 ± 0.61
TDACAPS [25] + FE	Squash [14]	84.77 ± 0.82	81.90 ± 1.09
TDACAPS [25]+FE	e-Squash	85.46 ± 0.92	77.23 ± 0.41
FFiCAPS + FF	Squash [14]	81.74 ± 1.53	78.07 ± 0.92
FFiCAPS + FF	HSquash [22]	82.06 ± 3.51	78.15 ± 1.17
FFiCAPS + FF	Strict-squash [23]	82.71 ± 1.66	75.95 ± 0.87
FFiCAPS + FF	Squash-4 [24]	82.39 ± 1.29	77.52 ± 0.86
FFiCAPS + FF	e-Squash	**86.58** **±** **2.70**	**82.12** **±** **0.90**

Bolded fonts stand for best performance in each column.

**Table 7:** Training time and recognition time for all methods.

Methods	Training time for electrode displacement (s)	Training time for different subjects (s)	Recognition time (ms)
SVM + FE [18]	0.08 ± 0.00	64.68 ± 4.03	0.036 ± 0.001
RF + FE [19]	0.81 ± 0.03	46.76 ± 2.54	0.014 ± 0.001
CNN [20]	90.21 ± 3.96	533.32 ± 16.18	0.128 ± 0.004
CNN + FE	26.98 ± 0.53	146.91 ± 4.51	0.075 ± 0.002
CNN + FF	33.14 ± 0.46	189.89 ± 0.92	0.095 ± 0.003
DNN + FE [21]	17.18 ± 0.29	88.90 ± 0.77	0.057 ± 0.003
TDACAPS [25]	214.77 ± 6.36	1980.31 ± 13.39	1.076 ± 0.030
CAPS + FF	213.20 ± 4.00	1971.36 ± 10.25	1.186 ± 0.079
*∗*FFiCAPS	221.31 ± 5.99	2079.93 ± 9.27	1.143 ± 0.083

## Data Availability

The data used to support the findings of this article are available from the corresponding author upon reasonable request.

## References

[1] Liu X., Xi X., Hua X., Wang H, Zhang W (2020). Feature extraction of surface electromyography using wavelet weighted permutation entropy for hand movement recognition. *Journal of Healthcare Engineering*.

[2] Li K., Zhang J., Wang L., Zhang M., Li J., Bao S. (2020). A review of the key technologies for sEMG-based human-robot interaction systems. *Biomedical Signal Processing and Control*.

[3] Li X., Wang S., Zhang Y., Wu Q. (2021). Hand motion recognition via multi-kernel manifold learning. *Journal of Ambient Intelligence and Humanized Computing*.

[4] Xue Y., Ju Z. SEMG based intention identification of complex hand motion using nonlinear time series analysis.

[5] Duan F., Ren X., Yang Y. (2021). A gesture recognition system based on time domain features and linear discriminant analysis. *IEEE Transactions on Cognitive and Developmental Systems*.

[6] Oh S. L., Hagiwara Y., Raghavendra U. (2020). A deep learning approach for Parkinson’s disease diagnosis from EEG signals. *Neural Computing & Applications*.

[7] Geng W., Du Y., Jin W., Wei W, Hu Y, Li J (2016). Gesture recognition by instantaneous surface EMG images. *Scientific Reports*.

[8] Chen L., Fu J., Wu Y., Li H., Zheng B. (2020). Hand gesture recognition using compact CNN via surface electromyography signals. *Sensors*.

[9] Barron O., Raison M., Gaudet G., Achiche S. (2020). Recurrent Neural Network for electromyographic gesture recognition in transhumeral amputees. *Applied Soft Computing*.

[10] Liu J.-w., Gao F., Lu R.-k. DDRM-CapsNet: capsule network based on deep dynamic routing mechanism for complex data.

[11] Cheng Y., Li G., Yu M. (2021). Gesture recognition based on surface electromyography-feature image. *Concurrency and Computation: Practice and Experience*.

[12] Phinyomark A., Phukpattaranont P., Limsakul C. (2012). Feature reduction and selection for EMG signal classification. *Expert Systems with Applications*.

[13] Phinyomark A., Hirunviriya S., Limsakul C., Phukpattaranont P. Evaluation of EMG feature extraction for hand movement recognition based on Euclidean distance and standard deviation.

[14] Sabour S., Frosst N., Hinton G. E. Dynamic routing between capsules.

[15] Ha K. W., Jeong J. W. Decoding two-class motor imagery EEG with capsule networks.

[16] Liu Y., Ding Y., Li C. (2020). Multi-channel EEG-based emotion recognition via a multi-level features guided capsule network. *Computers in Biology and Medicine*.

[17] Junior J. J. A. M., Freitas M. L. B., Siqueira H. V., Lazzaretti A. E., Pichorim S. F., Stevan S. L. (2020). Feature selection and dimensionality reduction: an extensive comparison in hand gesture classification by sEMG in eight channels armband approach. *Biomedical Signal Processing and Control*.

[18] Bian F., Li R., Liang P. SVM based simultaneous hand movements classification using sEMG signals.

[19] Wang F., Zhou J., Lin J., Wang H., Wang W., Yang J. A comparative study on sign recognition using sEMG and inertial sensors.

[20] Oh D.-C., Jo Y.-U. (2021). Classification of hand gestures based on multi-channel EMG by scale Average wavelet transform and convolutional neural network. *International Journal of Control, Automation and Systems*.

[21] Mukhopadhyay A. K., Samui S. (2020). An experimental study on upper limb position invariant EMG signal classification based on deep neural network. *Biomedical Signal Processing and Control*.

[22] Adu K., Yu Y., Cai J., Owusu‐Agyemang K., Twumasi B. A., Wang X. (2021). DHS‐CapsNet: d. *International Journal of Imaging Systems and Technology*.

[23] Chang S., Liu J. (2020). Multi-lane capsule network for classifying images with complex background. *IEEE Access*.

[24] Hollósi J., Á B. Training capsule networks with various parameters.

[25] Chen G., Wang W., Wang Z., Liu H., Zang Z., Li W. (2020). Two-dimensional discrete feature based spatial attention CapsNet for sEMG signal recognition. *Applied Intelligence*.

